RETRACTED

# SUMOylation of Mouse p53b by SUMO-1 Promotes Its Pro-Apoptotic Function in Ovarian Granulosa Cells

**DOI:** 10.1371/journal.pone.0063680

**Published:** 2013-05-16

**Authors:** Xiao-Ming Liu, Fei-Fei Yang, Yi-Feng Yuan, Rui Zhai, Li-Jun Huo

**Affiliations:** Key Laboratory of Agricultural Animal Genetics, Breeding and Reproduction, Education Ministry of China, College of Animal Science and Technology, Huazhong Agricultural University, Wuhan, People’s Republic of China; Institute of Zoology, Chinese Academy of Sciences, China

## Abstract

Follicular atresia is a process of spontaneous degradation of follicles, hindering growth and development in the mammalian ovary. Previous studies showed that follicular atresia was caused by apoptosis of granulosa cells, for which a number of apoptosis-related genes have already been identified. The roles of p53 in apoptosis of mouse granulosa cells and its post-translational modification are still unclear. The main objective of this study was to explore the roles of p53 in mouse granulosa cells. We found that mouse p53b, but not p53a, could be SUMOylated by SUMO-1 at lysine 375, which was essential for the protein stability of p53b in a dose-dependent manner. Immunofluorescent staining showed that wild p53b was located in the nucleus of granulosa cells, while its mutation of SUMOylated site (K375R) was localized in both nucleus and cytoplasm, implying that SUMOylation was necessary for the nuclear localization of p53b in granulosa cells. Overexpression of wild-type p53b, but not the mutation of SUMOylation site (K375R), significantly induced the expression of apoptosis-related gene, *Bax*, and increased the level of apoptosis in granulosa cells. This suggested that SUMO-1 modification of p53b was essential for inducing apoptosis in granulosa cells. Our results provide strong evidences that modification of p53b by SUMO-1 at lysine 375 was necessary for its activity to induce apoptosis in mouse granulosa cells, and it was involved in the regulation of p53b protein stability and nuclear localization. This implies that modification of p53b by SUMO-1 might regulate follicular atresia by inducing the apoptosis of ovarian granulosa cells in mice.

## Introduction

During the process of follicular atresia, follicles spontaneously degrade in the mammalian ovary, hindering growth and development. More than 99% of follicles disappear, primarily due to apoptosis of granulosa cells [1]–[6]. Although atresia can occur at any time during follicular development, the majority of follicles become atretic during the early antral stage of development [7]. The transition from preantral to antral follicles occurs after the granulosa cells are exposed to gonadotropin. The gonadotropin initiates differentiation of the granulosa cells making them susceptible to apoptosis.

RETRACTED

Apoptosis in granulosa cells is characterized by nucleosome DNA fragmentation, cell shrinkage, membrane blistering, and the formation of apoptotic bodies [8]. Many apoptosis-related factors have been implicated in follicular atresia, including death ligands and receptors, intracellular pro- and anti-apoptotic molecules, cytokines, growth factors, and a number of apoptosis-related genes, including the p53 gene [9]–[11].

The p53 protein is an antiproliferative transcription factor that increases the rate of transcription of various genes involved in mitosis and apoptosis [9], [12]–[15]. It plays a critical role in cell cycle regulation (G1/S transition), DNA repair, and induction of apoptosis [14], [16]–[18]. In granulosa cells, p53 content is correlated with contents of Fas and FasL, death ligands that are involved in the induction of apoptosis and are regulated by gonadotropins [19]. When gonadotropin induced, p53 becomes markedly elevated, suggesting that induction of atresia is p53-dependent [20]. Furthermore, overexpression of p53 resulted in increased Fas content and apoptosis [16]. However, mouse p53 gene contains only a promoter, which differs from the selective promoter of the human p53 gene; the alternatively spliced RNA species of tumor-suppressor gene p53 (which contains an additional 96 bases derived from intron 10) is present at approximately 25 to 30% the level of regularly spliced p53 RNA in both normal epidermal cells, carcinoma cells, and mouse liver and testis cells [21]. Precisely because of this alternative splicing, there are two types of p53 protein: p53a encodes 390 amino acids and p53b encodes 381 amino acids. The main difference between p53a and p53b is the C-terminal sequence. However, the biological properties of different types of the p53 protein in mice have not yet been determined.

The half-life of the p53 protein in normal cells is increased when the cells are exposed to various kinds of external stimuli. These stimuli influences the post-translational events and the stability of the protein, including acetylation, methylation, phosphorylation, ubiquitination, neddylation, and SUMOylation [22]–[24]. The small ubiquitin-related modifier-1 (SUMO-1) is an ubiquitin-related protein that was discovered in the yeast *Saccharomyces cerevisiae* in 1995 [25], [26]; SUMO-1 is involved in many cellular processes, including cell proliferation, differentiation, and apoptosis [25], [27]. Studies have reported that human p53 can be modified by SUMO-1 and the SUMOylation site is lysine386 [28]–[30]. Conjugation of SUMO-1 to wild-type p53 results in an increased transactivation ability of p53 [28], [30]. However, SUMOylation has no effect on mutant p53 transcriptional activity [29], [31]. In addition to comparing wild-type and SUMOylation-deficient p53 for transactivation, studies analyzed potential differences in localization and growth inhibition or apoptosis. Mutating the p53 SUMO-acceptor site lysine386 to arginine had no obvious effect on p53 localization [29], but one study generated p53-SUMO-1 fusion protein as a model for the effect of SUMO modification on the localization and function of p53, showing that p53-SUMO-1 fusion protein significantly redistributed from the nucleus to the cytoplasm when the SUMOylation site lysine386 was destroyed [32]. Studies showed the SUMOylation of p53 enhanced the apoptosis in Saos-2 cells [33]. In addition, SUMO modification of *Drosophila* p53 is required for its pro-apoptotic activity [34].

RETRACTED

While it is not very clear whether p53 is involved in regulating follicular atresia and granulosa cells apoptosis, and its regulatory mechanism is also unclear. Furthermore, there are two types of p53 protein (p53a and p53b) in mice, and the roles of these p53 forms in mouse granulosa cells and whether they can be SUMOylated have not been reported. In this study, the main objective is to explore the roles of p53 in mouse granulosa cells and the effects of SUMOylation.

## Materials and Methods

### Experimental Animals

We obtained immature 21 to 23 d-old Kunming White female mice from the Centre of Laboratory Animals of Hubei Province (Wuhan, PR China). All animal treatment procedures were approved by the Ethical Committee of the Hubei Research Center of Experimental Animals (Approval ID: SCXK (Hubei) 2008-0005). Mice were housed under controlled temperature (24°C) and lighting (12 h light/12 h darkness) with food and water ad libitum. Follicle development was primed by injection of each mouse with 10 IU pregnant mare serum gonadotropin (PMSG; SanSheng, Ningbo), and mice were killed by cervical dislocation 44–48 h later.

### Plasmid Construction

A 1310-bp mouse p53a and a 1213-bp mouse p53b cDNA sequence were amplified using polymerase chain reaction (PCR) from mouse ovary cDNA using the following primers: p53a- Forward 5′-CGGGATCCGGCAGGGTGTCACGCTTCT-3′; p53a- Reverse 5′-CGGAATTCCG AGGGACCGGGAGGATTGT-3′; p53b- Forward 5′-CGGGATCCGGCAGGGTGTCACGCTTCT-3′; and p53b- Reverse 5′- GCGAATTCGGAGGGATGAAGTGATGGGA-3′. Both included BamHI and EcoRI restriction sites. We subcloned into pCMV-N-HA to generate a HA-tagged p53a and p53b cDNA.

To generate the p53b lysine 375 arginine mutant, two pairs of primers were used for PCR: Pair 1- Forward 5′- CGGGATCCGGCAGGGTGTCACGCTTCT-3′; Pair 1- Reverse 5′- GGGCTTTCCTCCCTGATCAAGGCTTGG -3′; Pair 2- Forward 5′- CGGGATCCGGCAGGGTGTCACGCTTCTCCGAAGACTGGATT-3′; and Pair 2- Reverse 5′-GCGAATTCGGAGGGATGAAGTGATGGGAGCTAGCAGTTTGGGCTTTCCTCCCTG -3′. Amino acid of p53b was mutated from lysine to arginine using the p53b cDNA sequence as the template for the first reaction and the product as the template for the second reaction. The results were confirmed by sequencing.

RETRACTED

HA-tagged sumo-1 or ubc9, or Flag-tagged sumo-1 was preserved in our laboratory.

### In vitro Culture of Granulosa Cells and DNA Transfection

Granulosa cells from pre-ovulatory follicles (pre-GCs) were obtained from ovaries of 21 to 23 d-old Kunming White female mice injected with 10 IU PMSG (SanSheng, Ningbo) 44–48 h. Granulosa cells were cultured in 6-well culture plates in Dulbecco’s Modified Eagle’s Medium/Nutrient F-12 (DMEM/F12; Gibco) medium with 10% fetal bovine serum (FBS; Invitrogen), 60 mg/mL penicillin, and 50 mg/mL streptomycin. All cultures were maintained in DMEM/F12 medium at 37°C in a humidified atmosphere of 5% CO_2_. After being cultured 24 h, granulosa cells were washed by phosphate-buffered saline (PBS), and cultured for 24 h in fresh serum-free DMEM/F12 medium before DNA transfections.

For DNA transfection or co-transfection, granulosa cells were plated and then transfected with 4 µg of the desired plasmids for 24 h with Lipofectamine LTX (Invitrogen) according to manufacturer’s instructions. Desired plasmids and LTX were diluted in Opti-MEM (Gibco) medium and incubated for 5 min. This solution was then mixed with granulosa cells at a proportion of 1∶1.5 for 30 min; 24 h after transfection, granulosa cells were collected for protein extraction or apoptosis analysis.

To study the effect of SUMO-1 mediated modification of p53b on its protein level in granulosa cells, different dosages of pCMV-Flag-sumo-1 plasmids (2 µg, 3 µg, 4 µg, and 6 µg) were co- transfected with a fixed proportion of pCMV-HA-p53b or pCMV-HA-p53b^K375R^ (2 µg) plasmids into granulosa cell.

### Protein Extraction, Immunoprecipitation and Western Blot Analysis

Subconfluent cells seeded on 6-well culture plates were transfected with the expression vectors indicated. At 24 h after transfection, cells were washed twice with ice-cold PBS and harvested in 80 µL of ice-cold RIPA buffer (Santa Cruz), containing 10 µM phenylmethylsulfonyl fluoride (PMSF; DingGuo, Beijing) and 10 mg/mL protease inhibitors cocktail (Santa Cruz). Protein lysis was performed on ice for 20 min. Then, the lysates were centrifuged at 12000 rpm for 5 min, and the supernatant was collected and stored at −80°C.

The concentration of total protein was determined by bicinchoninic acid (BCA) assay (Pierce, Rockford, USA), and 20 µg of total protein was subjected to gel electrophoresis. The cell lysates mixed with 2× SDS gel-loading buffer were loaded on 4% stacking gel and 10% separating gel, and were then transferred to 0.2 µm polyvinylidene fluoride (PVDF) membrane (Milli-pore, Bedford, MA). After blocking in TBST [10 mM Tris (pH 7.5), 150 mM NaCl and 0.05% Tween 20] containing 5% skimmed milk (Sigma-Aldrich), membranes were incubated with the corresponding primary antibody diluted in blocking buffer overnight at 4°C. Polyclonal rabbit anti-p53 IgG (1∶500 dilution; Boster, Wuhan), monoclonal mouse anti-β-actin IgG (1∶500 dilution; Santa Cruz), and monoclonal mouse anti-HA IgG (1∶750 dilution; CWBIO, Beijing) were used as the primary antibody, respectively. After incubation with the primary antibody, the membrane was washed three times in TBST, and incubated with HRP-conjugated secondary antibodies diluted in TBST for 1 h at room temperature, then washed three times in TBST. Chemiluminescent detection was performed using ECL Western blot detection reagents (Amersham Biosciences, Piscataway, NJ). To analyze the SUMO-1 modification of p53 protein, membranes were probed with the HA antibody or p53 antibody, respectively, while the membrane was probed with β-actin antibody for normalization. The band intensities were measured with Gel-Pro analyzer 4.0 (Media Cybernetics, USA).

RETRACTED

Immunoprecipitation (IP) was conducted to detect if p53 could be modified by SUMO-1 in granulosa cells in vivo. Briefly, after transfection with pCMV-Flag-sumo-1 plasmid or pCMV-Flag plasmid (as a negative control), granulosa cells (10^6^−10^7^) were harvested in 1 mL lysis buffer (50 mM Tris HCl, pH 7.4, 150 mM NaCl, 1 mM EDTA, 1% Triton X-100) containing 10 µM PMSF (DingGuo, Beijing) and 10 mg/mL protease inhibitors cocktail (Santa Cruz). The extract was centrifuged at 12,000 g for 15 min at 4°C, and the supernatant were collected. 800 ul of the supernatant were incubated with ANTI-FLAG M2 Affinity beads (Sigma-Aldrich) overnight at 4°C with continual shaking. After recovery by centrifugation at 8,000 g for 30 s, the beads were washed four times with ice cold TBS (50 mM Tris HCl, 150 mM NaCl, pH 7.4). Then Flag-fusion proteins were eluted by 100 µL 3× FLAG peptide (Sigma-Aldrich) at 4°C with gentle shaking for 30 min. After elution, the beads were centrifuged at 8,000 g for 30 s and the supernatant was collected. For Western blot, the supernatant was mixed with equal volume of 2× SDS loading buffer and heated for 5 min at 100°C before being loaded on a SDS-PAGE gel. Polyclonal rabbit anti-p53 IgG was used as the primary antibody.

RETRACTED

In order to confirm which type of p53 (p53a or p53b) could be modified by SUMO-1, granulosa cells were co-transfected with pCMV-Flag-sumo-1 plasmid and pCMV-HA-p53a plasmid or pCMV-HA-p53b plasmid. After transfection, Flag tagged SUMO-1 were pulled down by Flag antibody and then HA antibody were used to detect the expression of p53a or p53b by Western blot.

### Immunofluorescence Cytochemistry

In order to detect the subcellular localization pattern of p53b and p53b^K375R^, pre-GCs were plated on coverslips and transfected with pCMV-N-HA-p53b or pCMV-N-HA-p53b^K375R^ vector respectively. After 24 h transfection, cells were washed twice with PBS and were fixed in 4% paraformaldehyde (Santa Cruz) for 15 min. Next, the cells were washed in PBS three times and then permeabilized in PBS containing 0.5% Triton-100 (Santa Cruz) at room temperature for 20 min. After blocking in PBS containing 5% bovine serum albumin (BSA) (Santa Cruz), cells were washed in PBS three times. After that, cells were incubated with anti-HA primary antibody (1∶100 dilution, CWBIO, Beijing) at 37°C for 2 h, followed by FITC-conjugated secondary antibody (1∶100 dilution, Boster, Wuhan) in the dark. The nucleus of cells was stained in 10 µg/mL propidium iodide (PI; Santa Cruz) for 5 min. Slides were mounted in DABCO (Sigma-Aldrich,) and viewed under a Zeiss- LSM 510 Meta confocal microscope.

For co-localization study of p53b or p53b^K375R^ with SUMO-1 in granulosa cells, pre-GCs were co-transfected with pCMV-Flag-sumo-1 plasmid and pCMV-HA-p53b plasmid or pCMV-HA-p53b^K375R^ plasmid. After 24 h transfection, SUMO-1 and p53b or p53b^K375R^ were detected by polyclonal rabbit anti-SUMO-1 antibody (1∶200 dilution; Santa Cruz) or monoclonal mouse anti-HA antibody (1∶100 dilution, CWBIO, Beijing), respectively. Cy3-conjugated anti-rabbit IgG antibody (1∶100 dilution, Boster, Wuhan) or FITC-conjugated anti-mouse IgG antibody (1∶100 dilution, Boster, Wuhan) were used as the secondary antibody, respectively. The nucleus was stained in 10 µg/mL 4′,6′,-diamidino-2-phenylindole (DAPI; Santa Cruz).

### Cell Apoptosis Assay

Pre-GCs were transfected with pCMV-N-HA-p53b, pCMV-N-HA-p53b^K375R^, or negative control pCMV-N-HA for 24 h. Cells were washed twice in PBS, then trypsinized and collected for apoptosis assay. Apoptosis was performed by using the AnnexinV kit (AntGene, Wuhan) according to manufacturer’s instructions. Cells were incubated in AnnexinV–FITC and PI solution at room temperature in the dark for 15 min, then 300 µL of 1 × binding buffer was added to each sample. Flow cytometric analysis was conducted using a BD FACSCalibur (Becton, Dickinson and Company, USA; Ex, 488 nm and Em, 530 nm).

RETRACTED

### Real-time RT-PCR Analysis

To determine genes regulated by SUMOylation of p53b, at 24 h after transfection, total RNA was prepared using the RNAiso Plus (TaKaRa, Dalian), and in vitro transcription was carried out using PrimeScript RT reagent Kit With gDNA Eraser (TaKaRa, Dalian). Real-time PCR was then conducted to quantify the steady-state mRNA levels of the tested genes using SsoFast™ EvaGreen® Supermix (Bio-Rad, USA) on the Bio-Rad CFX96 Real-time PCR System. The threshold cycle (Ct) was used to determine the relative expression level of each gene by normalizing to the Ct of *β-actin* mRNA. The method of 2–ddCt was used to calculate the relative fold change of each gene. To ensure that only target-gene sequence-specific, non-genomic products were amplified by real-time PCR, careful design and validation of each primer pair, as well as cautious manipulation of RNA, were undertaken to quantify the steady-state mRNA levels of *Bax* and housekeeping gene *β-actin* (internal control). The primers used were *Bax-* forward: 5-CCAGGATGCGTCCACCAA-3; *Bax-* reverse: 5-CAAAGTAGAAGAGGGCAACCAC-3; *β-actin-* forward: 5- CCCATCTACGAGGGCTAT-3; and *β-actin-* reverse: 5-TGTCACGCACGATTTCC-3. Calculation of the relative fold change of *Bax* was done using the method of 2^−ΔΔCt^. In each experiment, levels of *Bax* mRNA were presented as relative changes to a specific group (control), in which its expression level was set at 1.

### Data Analysis and Statistics

All experiments were performed independently at least three times, and data are presented as mean ± SD. Differences between groups were analyzed by one-way ANOVA followed by Tukey’s Honesty Significant Difference (HSD) test using SPSS (Version 17.0; SPSS, Chicago, IL, USA). *P*<0.05 was considered significantly different, and *P*<0.01 was extremely significantly different.

## Results

### SUMOylation Increased the Expression Level of Mouse p53 Protein

At 24 h after transfection, total proteins were extracted from the cells and analyzed by Western blot using the HA-specific antibody or p53-specific antibody. After transfection with p53a or p53b plasmid, the expression of HA-p53 fusion protein or increased level of p53 protein could be observed (Fig. 1, lanes 3 and 4). Interestingly, after transfection with HA-sumo-1 or HA-ubc9 plasmid, a shifting-up band detected by using anti-HA antibody was also visible (Fig. 1, lanes 5 and 6), which was consistent with a form of protein that was covalently modified by HA-SUMO-1 or HA-UBC9. More importantly, the expression of p53 protein was significantly increased by transfection with sumo-1 or ubc9 plasmid (Fig. 1, lanes 5 and 6). Thus we predicted that the shifting band detected by HA antibody represented HA-SUMO-1-p53 fusion protein.

RETRACTED

**Figure 1:** SUMOylation increased the expression level of mouse p53 protein. Pre-GCs were seeded in 6-well culture plates and transfected with 2 µg of HA-p53a, HA-p53b, HA-sumo-1, HA-ubc9, or empty HA expression plasmids. 20 µg total extracts were prepared and resolved by SDS–PAGE and analyzed by Western blot using anti-HA (the top group) or anti-p53 (the middle group) specific antibody. Positions of molecular weight markers, free HA-p53 or putative p53/HA–SUMO-1 and p53/HA-UBC9 conjugates are indicated. β-actin is a loading control.

### SUMO-1 Conjugation to p53b in vivo Requires Lysine 375

Based on the results above, we speculated that the mouse p53 protein could also be modified by SUMO-1. Immunoprecipitation (IP) study was designed to confirm whether mouse p53 could be SUMO-1 modified or not in granulosa cells. Pre-GCs were transfected with pCMV-Flag-sumo-1 plasmid or pCMV-Flag plasmid (as a negative control) for 24 h. Flag-tagged protein were pulled down by anti-Flag affinity beads and then analyzed by Western blot using anti-p53 antibody. A visible band of p53 was observed in the sample of pCMV-Flag-sumo-1 transfected granulosa cells, but not in the control sample (Fig. 2A). This study clearly showed that mouse p53 protein could be SUMO-1 modified in granulosa cells in vivo. However, there are two types of p53 in mouse, and which type of p53 that could be modified was unknown. Previous studies showed lys386 of human p53 was required for SUMO-1 modification in Saos-2 cells [29], [35], [36]. To identify which type of mouse p53 could be modified by SUMO-1 in mouse, we aligned the protein sequence of mouse p53a and p53b to human p53 around the SUMOylation site at lys386 (Fig. 2B). The lysine 375 of 374IKEE377 in mouse p53b was aligned to the lysine within the consensus SUMOylation site of human p53, 385FKTE388 (Fig. 2B). The region 374IKEE377 of mouse p53b was also confirmed as a high probability SUMOylation site, with a score of 2.943 predicted by SUMOsp2.0.4 software. However, there are no conserved amino acids in mouse p53a with mouse p53b at lys375 or human p53 at lys386, and there are no SUMOylated sites in mouse p53a predicted by SUMOsp2.0.4 software. In order to further confirm if only p53b, but not p53a, could be SUMO-1 modified in granulosa cells, pre-GCs were co-transfected with Flag-tagged sumo-1 plasmid and HA-tagged p53a or p53b plasmid. After transfection, the Flag-tagged fusion protein were pulled down by Flag antibody and then detected by western blot using HA antibody. The results showed that only p53b, but not p53a, could be co-immunoprecipitated by Flag-tagged sumo-1 (Fig. 2C).

RETRACTED

**Figure 2:** Identification of SUMOylation of p53b in vivo at Lys 375. (A) Immunoprecipitation analysis of SUMOylation of p53 in vivo. Pre-GCs were transfected with pCMV-Flag-sumo-1 plasmid or pCMV-Flag plasmid. Flag-tagged protein were pulled down by anti-Flag affinity beads and then analyzed by Western blot using anti-p53 antibody. A visible band of p53 was detected in the sample of pCMV-Flag-sumo-1 transfected granulosa cells, but not in the control sample. (B) SUMOylation consensus site aligned in sequences of p53 from human and mouse. The SUMOylation consensus site is ψKXE with a hydrophobic residue, such as Phenylalanine (F), Isoleucine (I), or Leucine (L). Sequences of human p53 and mouse p53b were aligned. Lys386 in human p53 is SUMO-1 modified and the mouse p53b has a highly homologous sequence to this SUMOylation site. (C) Co-immunoprecipitation of SUMO-1 with p53a or p53b. Pre-GCs were co-transfected with Flag-tagged sumo-1 plasmid and HA-tagged p53a or HA-tagged p53b plasmid. Flag-tagged proteins were pulled down by anti-Flag affinity beads and then analyzed by Western blot using anti-HA antibody. A band of p53 (p53b) was detected in the sample of Flag-sumo-1 plasmid and HA-p53b plasmid co-transfected granulosa cells, but not in the HA-p53a plasmid and Flag-sumo-1 plasmid co-transfection group or control sample. (D) p53b is SUMOylated at lys375. Pre-GCs were co-transfected with 2 µg of wild type HA-p53b or mutant p53b (K375R) plasmid and 2 µg of Flag-sumo-1 plasmid. 20 µg total extracts were prepared and resolved by SDS–PAGE and analyzed by Western blot using the anti-HA-specific antibody. Positions of molecular weight markers, free p53 or p53-SUMO-1 conjugates are indicated. β-actin is a loading control. After transfection, two bands could be detected in the group with co-transfection of wild type p53b and sumo-1, the lower molecular weight below was considered as free p53b and the higher molecular weight above was p53b-SUMO-1 as the SUMOylated p53b, but only one band (mutant p53b) could be observed in the group with co-transfection of mutant p53b and sumo-1 plasmids, while the p53b (K375R)-SUMO-1- band was not observed.

Although Lys375 of p53b were predicted by SUMOsp2.0.4 software as a putative SUMO-1 modified site, it is still unknown whether this Lys375 is necessary for p53b’s modification by SUMO-1. Therefore, we mutated lysine 375 of mouse p53b to arginine and generated a mutant, HA-tagged p53b (K375R) expression plasmid. Wild-type p53b plasmid or mutant p53b plasmid, with sumo-1 plasmid, were co-transfected into mouse pre-GCs and analyzed by Western blot to examine the expression and SUMOylation. When cells were co-transfected with wild-type p53b plasmid and sumo-1 plasmid, two bands were detected (Fig. 2D, lane 3), but only one band could be observed when co-transfected with mutated p53b (K375R) plasmid and sumo-1 plasmid (Fig. 2D, lane 4). The lower band (55 kDa) was considered p53b protein and the band above was considered SUMO-1 covalently conjugated p53b protein, SUMOylated p53b. These results supported our hypothesis that mouse p53b could be SUMO-1 modified, and lysine 375 of p53b was necessary for SUMO-1 modification. The SUMOylation of mouse p53b at lys375 by SUMO-1 raised another interesting question: what regulatory roles of SUMOylation of p53b plays on the function of p53b in mouse ovarian granulosa cells. Further experiments were conducted to explore the effects of SUMOylation modification of p53b on its protein stability, subcellular localization, and biological activity in mouse granulosa cells.

RETRACTED

### SUMO-1 Modification Enhanced the Protein Stability of p53b in a Dose-dependent Manner

Our results above showed that transfection with sumo-1 or ubc9 plasmid could enhance the expression level of p53 in granulosa cells. To further explore the patterns of SUMO-1 modification to enhance the stability of p53b, pre-GCs were co-transfected with HA-wild-type p53b or HA-p53b (K375R) plasmid and different amounts of Flag–sumo-1 plasmids. Total proteins were extracted and subjected to Western blot analysis with HA antibody (Fig. 3). As predicted, increasing the amount of Flag-sumo-1 plasmid for transfection resulted in a significant increase of both SUMOylated p53b and free p53b in a dose-dependent manner (Fig. 3A and B, compare lanes 3, 4, 5, and 6), but did not increase p53b (K375R) (Fig. 3C). These results demonstrated that SUMO-1 modification was responsible for increasing the stability of p53b in a dose-dependent manner, and further confirmed that Lys 375 was required for SUMOylation of p53b by SUMO-1.

**Figure 3:** SUMO-1 modification enhanced the stability of p53b in a dose-dependent manner. (A) Pre-GCs were co-transfected with 2 µg HA-p53b plasmid and different amounts (2 µg, 3 µg, 4 µg, and 6 µg) of Flag-sumo-1 plasmids. 20 µg total proteins were prepared and resolved by SDS–PAGE and analyzed by Western blot using anti-HA-specific antibody. Positions of molecular weight markers, free p53b and p53b-SUMO-1 conjugates are indicated. β-actin is a loading control. (B) Relative expression quantity of p53b and SUMO-1-p53b were determined by densitometric scans. The total amount of β-actin present in the lower set of lanes was used to standardize the amount of p53b and SUMO-1-p53b present in the upper set of lanes. The value expressed by each bar represents the mean ± SD (n  = 3). Different letters indicated statistical difference (*P*<0.05). (C) Pre-GCs were co-transfected with 2 µg HA-p53b (K375R) and different amounts (2 µg, 3 µg, 4 µg, and 6 µg) of Flag-sumo-1 plasmids. HA antibody were used to detect the expression of p53b (K375R) after transfection. The results showed that elevating the amount of transfected Flag-sumo-1 resulted in a simultaneous increase in the level of SUMOylated p53b and free p53b, but not mutant p53b (K375R).

RETRACTED

### SUMO-1 Modification was Required for the Nuclear Accumulation of p53b in Granulosa Cells

In order to study whether SUMO-1 modification of p53b at Lys375 is involved in the regulation of p53b’s subcellular localization in granulosa cells, pre-GCs were transfected with HA-p53b plasmid or mutant HA-p53b (K375R) plasmid, immunofluorescence cytochemistry was used to detect the subcellular localization of p53b protein by HA antibody. Wild type p53b proteins were accumulated only in the nucleus of pre-GCs, while mutant p53b (K375R) were localized in both nucleus and cytoplasm of pre-GCs (Fig. 4A). Meanwhile, the co-localization of SUMO-1 with p53b was observed in the nucleus of granulosa cells after co-transfection with sumo-1 plasmid and p53b plasmid. Mutant p53b (K375R) was still localized in both nucleus and cytoplasm of granulosa cells after co-transfection with sumo-1 plasmid and p53b (K375R) plasmid. Overall, the results indicated that SUMO-1 modification of p53b at Lys 375 was required for its nuclear accumulation in mouse granulosa cells.

**Figure 4:** SUMO-1 modification of p53b at Lys 375 was required for its nuclear accumulation in granulosa cells. (A) Pre-GCs were transfected with HA-tagged p53b or mutant p53b (K375R) plasmid, respectively. Then immunofluorescence cytochemistry was used to detect the subcellular localization of p53b or p53b (K375R) by HA antibody. The immunostaining signal of p53b were observed in nucleus of granulosa cells, but p53b (K375R) were seen in both nucleus and cytoplasm of granulosa cells (green). The nucleus was stained by PI (red). (B) Pre-GCs were co-transfected with HA-tagged p53b or mutant p53b (K375R) plasmid with Flag-tagged sumo-1 plasmid. Wild type p53b and mutant p53b (K375R) were detected by HA antibody with FITC-conjugated secondary antibody (green) and SUMO-1 was detected by SUMO-1 antibody with Cy3-conjugated secondary antibody (red), and the nucleus was stained by DAPI (blue). Co-localization of SUMO-1 and p53b in the nucleus were observed, but p53b (K375R) were still localized in both nucleus and cytoplasm of granulosa cells.

### p53b-induced Cell Apoptosis was Enhanced by SUMO-1 Modification

As p53 is a cellular gatekeeper [14], [37], one of its roles is to survey cellular stress and induce apoptosis, if necessary. Therefore, we investigated the roles of mouse p53b in inducing apoptosis of pre-GCs. Cells were transfected with wild-type p53b or mutant p53b (K375R) for 24 h and then collected for apoptosis analysis by flow cytometer. The apoptosis rate was significantly increased by transfection with wild-type p53b compared with the control group and mutant p53b (K375R; Fig. 5A and 5B; *P*<0.05). The mutant p53b (K375R) transfected cells also showed significant increases in apoptosis compared with the control group (*p*<0.05), but were significantly lower in apoptosis compared with wild p53b transfected group (*p*<0.05). In addition, RT-PCR was used to detect the expression of a marker of apoptosis (*Bax*). Overexpression of either wild type p53b or mutant p53b (K375R) could significantly increase the expression of *Bax* mRNA, compared with control group. However, overexpression of wild type p53b could induce much higher expression level of *Bax* mRNA, compared with mutant p53b (Fig. 5C). These results were consistent with our other findings related to the apoptosis rate of granulosa cells. All these results implied that SUMO-1 modification of p53b enhanced the ability of p53b to induce apoptosis in pre-GCs. Mutating the SUMOylation site of p53b could significantly weaken the activity of p53b to induce apoptosis and apoptosis-related gene, *Bax*. On the other hand, in addition to inducing apoptosis, the cell death ratio was increased by mutation of p53b (K375R), but not by wild-type p53b (Fig. 5A).

RETRACTED

**Figure 5:** SUMOylation of p53b induced apoptosis in granulosa cells. (A) Representative flow cytometric analysis of apoptotic cells stained with Annexin V-FITC and PI after transfection with 2 µg wild type p53b, mutant p53b (K375R) plasmid, control plasmid or non-transfection control group for 24 h. In each panel, the lower right quadrant contains apoptotic cells (positive for Annexin V and negative for PI). (B) The apoptosis rate of granulosa cells. The value expressed by each bar represents the mean ± SD (n = 3). Different superscripts denote statistical difference at a *P*<0.05. (C) Expression level of *Bax* mRNA. 24 h after transfection with 2 µg wild type p53b, mutant p53b (K375R), control plasmid or non-transfection control group, expression level of *Bax* mRNA was detected by quantitative real-time PCR. Fold changes were calculated from *β-actin* normalized Ct values. The value expressed by each bar represents the mean ± SD (n = 3). Different superscripts denote statistical difference at a *P*<0.05.

## Discussion

In normal cells, p53 is maintained at a low level, which is partly due to the short half-life of the protein [38]. However, in response to a variety of stress signals, p53 is stabilized, causing protein to accumulate and activating p53-dependent transcription. Related factors, including lower levels of the MDM2-mediated poly-ubiquitination of p53 and others, improved post-translational modifications [22]–[24].

RETRACTED

Although human p53 had been reported to be modified by SUMO-1 [11], [28], [39], there are two kinds of p53 (p53a and p53b) in mouse; whether mouse p53 could be SUMOylated was unclear. In this study, overexpression of sumo-1 or ubc9 could increase the protein level of p53 in granulosa cells, and a specific migrating band was also observed by using HA antibody, implying that SUMOylation is involved in the stability of p53 protein by post-translational modification. Based on the prediction results of SUMOsp2.0.4 software, there is a conserved SUMOylated site at lys375 of p53b, but not in p53a. The results of IP confirmed that mouse p53b, but not p53a, could be SUMO-1 modified at lys375. Further experiments showed that lys375 mutation of p53b could result in its nucleus-cytoplasm translocation and decrease its ability to induce apoptosis, confirming that p53b modified at lys375 by SUMO-1 plays crucial roles for p53 functions in granulosa cells.

The SUMO-1 modification increased the stabilization of mouse p53b in a dose-dependent manner (Fig. 3A); these results were similar to the results in U20S cells, in which SUMO-1 modified form of p53 accumulated after UV irradiation [36]. However, several researchers have delineated a conserved pathway, in which SUMOylation and ubiquitination cooperate in protein degradation [40]. Topors is an ubiquitin and small ubiquitin-like modifier ubiquitin-protein isopeptide ligase (SUMO E3) ligase [41]. Polo-like kinase 1 (Plk1) mediated phosphorylation of Topors inhibited Topors-mediated SUMOylation of p53, whereas p53 ubiquitination was enhanced, leading to p53 degradation [42], whether SUMOylation and ubiquitination of p53 cooperate in its degradation or the SUMOylation of p53 enhances the stabilization of p53 is still unclear. One research group proposed a hypothesis about an involvement of SUMOylation in p53 degradation [43], while there was some experimental evidences that SUMOylation may indeed facilitate p63 and p73 degradation [44], [45]. Considering that in our results, the stabilization of p53b was increased by SUMOylation (perhaps because it prevented ubiquitination), SUMOylation of p53b may inhibit its degradation by competing for the same lysine residue that was required for p53 ubiquitination or by interfering with conjugation of ubiquitin molecules to neighboring sites [46]. However, further studies will be required to address this issue.

RETRACTED

Another issue to be addressed is the role of the SUMO-1 modification pathway in the subcellular distribution of p53b. In normal cell circumstances, p53 protein is present in the nucleus, and p53 nuclear export is critical to determine their degradation; we can speculate that the distribution of p53 in the nucleus and cytoplasm is a key factor in determining its stability. Interestingly, it has been reported that p53-SUMO-1 fusion protein localize to PML bodies. While damages the use of the fusion proteins by mutating the C-terminal glycines in the SUMO-1 portion (ΔGG) to inhibit the formation of isopeptide bonds between SUMO-1 and target lysines, the localization of p53-SUMO-1ΔGG is predominantly at the nuclear envelope with some cytoplasmic staining [32]. Similarly, SUMOylation helped recruit *Drosophila* p53 to nuclear dot-like structures that could be marked by human PML and the *Drosophila* homologue of Daxx [34]. In our study, we also found that the localization of p53b was in the nucleus; after mutation, the nucleus localization was lost compared to wild p53b and part of the p53b was localized in the cytoplasm (Fig. 4 A and B). So our results directly demonstrated that SUMOylation was required for the nuclear localization of p53b, which provided a novel platform for explaining why the SUMOylation of p53b increased its stabilization.

Research has firmly established that p53, is the cellular gatekeeper for growth, division, apoptosis, tumor suppression, and reproductive regulation [14], [38], [47]. Loss of the p53 gene in female mice leads to a significant decrease of fertility. The p53 gene product regulates maternal reproduction at the implantation stage of the embryo [48]. In addition, p53 is required for the induction of apoptosis [49]. Apoptosis of granulosa cells is an essential component of ovarian follicular atresia [50], and it has been reported that p53 protein is mainly expressed in the apoptotic granulosa cells of atretic follicles in the ovary [51], [52] and p53 decreases the expression of the apoptosis-suppressing gene bcl-2 while simultaneously increased the expression of *Bax*, a gene that encodes a dominant inhibitor of bcl-2 protein [53], [54]. Previous studies had shown that human p53 could be SUMO-1 modified, and when mutated the SUMOylation site lys386, the ability of p53 to induce apoptosis was weakened or even disappeared [33]. Mutation of both SUMOylation sites of *Drosophila* p53 dramatically reduced the transcriptional activity of p53 and its ability to induce apoptosis in transgenic flies [34]. In our study, SUMOylation of p53b enhanced the apoptosis in pre-GCs; mutating the SUMOylation site of p53b could significantly weaken the activity of p53b in inducing cells apoptosis (Fig. 5A and 5B). Actually, we also tested the effect of sumo-1 or p53/sumo-1 co-transfection on apoptosis of granulosa cells, the results showed that sumo-1 transfection could also induce apoptosis of granulosa cells, but co-transfection with both p53 and sumo-1 has much more significant effect of inducing apoptosis of granulosa cells (data not shown). Meanwhile, overexpression of p53b significantly increased the expression of *Bax* (Fig. 5C). Interestingly, destruction of the SUMOylation site simultaneously decreased the expression of *Bax* (Fig. 5C). To some extent, p53b was regulated by SUMO-1 modification at the transcriptional level. However, further studies will be required to address whether SUMO-1 modification could enhance mouse p53b-dependent transactivation. Moreover, FSH is a potent survival factor of granulosa cells during follicular development. The future study about how FSH affects the SUMOylation of p53b-induced apoptosis during folliculogenesis will help us in better understanding of follicular development.

RETRACTED

In conclusion, our data demonstrated that mouse p53b, but not p53a, can be SUMO-1 modified, and the SUMOylation site is lys375. The SUMOylation modification is clearly important for the functions of mouse p53b, regulating its stabilization, nucleus-cytoplasm translocation, and pro-apoptosis ability. These results provide important information about the roles and regulatory pathways of p53 in follicular granulosa cell apoptosis, follicular atresia, and ovarian cancer.
